This article has been retracted.

# An Architectural Framework for Healthcare Dashboards Design

**DOI:** 10.1155/2021/1964054

**Published:** 2021-10-27

**Authors:** Saeed Rouhani, Shooka Zamenian

**Affiliations:** ^1^Faculty of Management, University of Tehran, Tehran, Iran; ^2^Mehr Alborz University, Tehran, Iran

## Abstract

In today's competitive environment, one of the new tools in the field of information technology is business or organizational dashboards that are a backup in the process of strategic management of organizations. The purpose of the current research is to provide a framework to design the healthcare dashboard through technical architecture with fulfilling the decision-makers' requirements. In this study, a common qualitative research method, metasynthesis, is applied, including a seven-step set of research questions, conducting systematic literature search and selection of suitable papers, data extraction, analysis and findings of the qualitative composition, quality control, and presentation of findings. During this process, 102 articles were found by saturation of information resources and then 12 articles were selected for extracting data using acceptance and rejection criteria. A critical evaluation method was used to evaluate the quality of selected articles. After investigating the selected articles and scoring them, in terms of quality, one article was very good, 10 articles were good, and one article was moderate. Then, with regard to the principles and guidelines of technical architecture, the required information was extracted from the selected articles and was analyzed with the method of open, axial, and selective coding. Following the steps of metasynthesis methods, the principles extracted with major and minor titles principles and guidelines in the form of multilayered system architecture including presentation layer, application layer, data layer, and technical infrastructure layer were classified. In the obtained framework, 15 indicators as the main principles and 66 subcriteria as the subsidiary principles for the design and technical architecture of enterprise dashboards were identified.

## 1. Introduction

Today, intense competition has dominated in various businesses. Senior executives and middle managers in organizations need to decide faster and more accurately than before. It is obvious that achieving fast and accurate knowledge is necessary for decision-making and consequently effective tools such as management dashboards are placed in the IT roadmap of firms [1]. Dashboards can be easily used as a tool to help evaluate performance and support efficient decision-making by identifying trends, patterns, and abnormalities to information [2]. It collects information accumulated from all sectors of the organization, which contains different resources related to a variety of business tasks. This information is incorporated and repeated by catering a user interface in the form of charts, reports, visual indicators, and alert mechanisms [2]. In the past, the dashboard was only used in different business segments; however, it has now been developed for other parts, such as a healthcare part [2]. Vilarinho et al. [3] have provided a more complete definition in his article; they presented the dashboard as a visual and interactive performance management tool that displays on the one screen the most important information to reach one or more individuals or organizational goals, allowing the user to identify, discover, and communicate problem areas that require reformative action. One of the functions of this tool is to promote everyone's participation in the process of improvement [3]. In their article [3], they pointed out that the dashboard has three basic objectives: (1) monitoring critical activities and processes by using alert criteria when performance is descended lower than the goals set, (2) analyzing the root causes of problems by using respective and timely presented information via multiple views and levels of detail, and (3) managing people and processes to improve decisions and direct the organization in the right direction [4].

Management dashboards are a subset of business intelligence systems, in fact, a new software system that helps organizations to enrich targets using information and analysis them. The dashboard is a total package of applications such as strategy maps, balanced scorecards, and business intelligence for performance management of organizations, which provide information on a specific format for decision-makers [5].

Hospital is a complex ecosystem of services, customers, personnel, equipment, data, and information that are produced in it [6]. In the past, hospital management was equal to financial management, but today with proper management, they can achieve integration between organizational intelligence (specialists), business intelligence (data types), and competitive intelligence (permanent communication with internal and external customers). This integration provides an opportunity for the hospital to have a view of the actual performance against strategic objectives and change to the innovative organization. Access to strategic information and timely for the correct and crucial decision is required to achieve this. To exchange such information and management priorities between different levels of operation using intelligent tools, dashboards can be very value-creating and effective [7]. Today, technological advances such as dashboards make it easier to access and easy to use and increase credit, and the integration of all clinical and environmental information in a single screen is made possible which improves worker productivity, accelerates decision-making and streamline workflow processes, and reduces negligence and errors in management and nursing performance [8].

Today, more integration of electronic health records (EHR) systems has made specialists of healthcare be able to retrieve approximately all health information via the computer. However, due to access to a large amount of data, information can be excessive and scattered, which can lead to the wasting of physicians' time to collect basic health information and the loss of crucial information that creates the field of medical errors [9]. But how to provide information due to the complexity and volume of them and the principles of design and technical architecture dashboard is very important, since decision-makers need to know how to provide the best information in real time so that they can make effective decisions. However, in recent years, a number of governmental agencies and NGOs have taken actions to create management dashboards, but they have limited success because, despite the popularity of the dashboard, there is little information about the principles and framework of making it to enhance the effectiveness. This means that the dashboard with which design and architecture will follow the best performance for the organization [10].

It is important that the quality of decision-making and achieving a high-performance organization depends on the quality of the information provided by the dashboard. Unfortunately, little research has been done in this regard and in production dashboards; the format of information presentation is opposed to visual techniques and has been mentioned very low to the ground of technical architecture of dashboards. The technical architecture of the dashboard is actually a general structure for its implementation based on a set of functional requirements of the system to be able to implement applications and dashboards quality to produce and keep it optimized and accelerated. Compliance with technical architecture can be expected to cover all technical and operational requirements [1, 10].

The dashboard in the health sector has two main roles, which include monitoring and performance evaluation process of healthcare organization, and also in the healthcare process; for this reason, the development of the healthcare dashboard has been considered for different sectors of healthcare and several studies have been done on it [2].

Thus, providing a framework for the design and architecting of organizational dashboards is an important and significant issue. The main question in this research that we have to respond to it is “what are the principles and guidelines for design and architecting of a convenient dashboard?” In this study, we try to provide a framework to design the healthcare dashboard through technical architecture with fulfilling the decision-maker's requirements. This study is structured in five parts: literature review, methodology, data analysis, discussion, and conclusions.

## 2. Literature Review

Generally, business intelligence and analytics (BI&A) term was applied to illustrate technologies [11, 12], analytical tools [13–15], systematic processes [16], methodologies [17], and techniques [18], which use computer-supported systems for collecting, analyzing, and propagating information for efficient business operations and better decision-making [19].

Business intelligence deals with a set of processes and software that support organizations in understanding business large datasets, retrieval and analysis of information, and decision. The value of graphical presentation of data is identified quickly in this field and it is usually in the form of a dashboard, interface similar to car dashboard that organizes the information and is easily displayed and read [20]. Business intelligence visualization dashboards provide a set of multiple visual components such as charts on a screen that information can be understood at a glance [21]. Beneficiaries in business intelligence systems involve a wide range of users including experts control, financial and financial affairs reporter, vendors, and board members [22]. Two prominent features of the new generation of business intelligence systems are integration and visualization. Dashboard reports key data of performance in the organization and integrated and real-time basic facilities. Dashboard, based on business intelligence systems, provides access to powerful analytical systems and tools in a user-friendly environment for managers. In addition, it helps to support analysis and decision-making throughout the organization [23].

With the development of dashboards, business intelligence tools have taken significant steps in the area of using electronic health records [24]. The most basic use of the dashboard platform is that it can integrate multiple data, data structures, and resources and display them in a single interface, which is easily displayed and understood, but providing real-time supervision of the health system's progress for personnel is the other benefits of the dashboard, which will enable key staffers to take reformative action [24]. With the full understanding of dashboards by health personnel, they can be answerable and do quick action to address any problems [24]. Efficiency, safety, and quality were the primary role of performance dashboards. However, dashboards utilization by health managers must be a sustainable process. [24].

There are many definitions for visualization. According to Card et al. [25], visualization is the use of visual presentations and interactive and data computers to increase understanding, where understanding means the power of human understanding or the acquisition or use of knowledge [26]. In fact, data visualization was designed to facilitate and decode intricate and vague data in graphical or visual formats for helping decision-makers to understand precisely difficult and ambiguous notions/ideas of them [27]. The main purpose of visualization is understanding insights [28].

Commonly, creation and studying of the visual representation of data is named data visualization, which is summarized in some schematic forms, containing features or variables, for the information sector to simplify the recognition of templates in the data [27]. The balanced scorecard (BSC) approach and the dashboard are two methods of the data visualization design, which are used for performance assessment, and they are appropriate for consequence appraisal [29, 30]. With graphical diagnostic abilities, which are complemented with colorful graphical indicators and easy-to-read measurement in the dashboard, organizations can able to monitor their improvement and recognize when it is necessary to change the path for ameliorating their performance [31].

Pérez-González et al. [32] argued that, for providing the feasibility of better representation of the consequence by applying visualizations and summarized tables, the dashboard application was developed and expanded. Dashboard design plays an important role in the decision-making process. Using the dashboard should be easy and includes capabilities such as personalization, targeting audience, and display in color in order to facilitate the decision-making process. Depending on the particular business, the design and features of the dashboard may be different [33]. Designers or technical architects must prepare the plan for infrastructure and provide characteristics of its components. Architects must pay attention to the present and future needs of the company and its expanding program. Technical architects in levels of the organization plan the company's overall infrastructure and create and publish standards about how different software is used [34].

After reviewing the research being undertaken in the field of principles of design and technical architecture for organizational dashboards, the mentioned indicators closer to the goal of our research were extracted through the research, and these indicators on the dashboard are near to the viewpoint of past researchers. In essence, the goal of designing a dashboard is to create transparency and accountability, which faces many risks challenges [35]. Hansoti [33] noted that the principles include displaying past data basis of date, data filtering capabilities, integration with data storage, visualization of data and personalization. These principles can be a guide for designing the public section dashboards more efficiently, and they can assist in improving dashboard design for creating transparency and accountability [35]. For example, the lack of updated, timely, and precise data contributed to misunderstanding and misinformation among citizens and decision-making managers [36].

Kuo et al. [37] point to four types of displaying information including timing, hierarchical, relational, and multidimensional and know that their results control and monitor the project using Gantt charts, ability to view the three-dimensional structure and its components and clear understanding of the organization and classification system for project control and achieve higher construction performance and understanding of the relationships between items and system components.

Lee et al. [9] said in their article that users for quick catch relevant information from a sophisticated system can get aid from the digital dashboard system which is a customary instance of a brief and specific text display system; in addition, it displays information on a large screen and led to increasing communication and information sharing.

For consciousness in healthcare or any other settings, using accessible data at an individual is not sufficient [38]. According to [39], “if data is not transmitted, absorbed, and assimilated in a timely procedure by the human to create situation consciousness, providing even one ton of data will not efficiently work.”

Pappas and Whitman [40] point to the possibility of comparing the data with line, bar, spot, scatter, bubble and charts. And also filtering and drilling down and viewing decrease and increase compared to the index using color sorting. The other aspect is grouping by the date or target group and know their results. In this manner, users achieve their goals faster and in more detail.

Elias and Bezerianos [41] point to principles such as possibility of grouping, drilling down, drilling up and filtering, and clear visual distinction between the data. Backward and forward moves, clipboard and labeling and writing notes for charts and lock for graphs, partial and total filtering, support for local language and provide detailed explanations about the functioning of buttons are necessary. Also they mentioned labels and icons available to users are crucial for dashboards. Also, beginners and experts can use partial or complete filter according to their needs, which caused good work for beginners who do not know about international terms of charts metrics and functions.

Ameliorating of the situation consciousness provided an understanding of main agents, to protect progress in the perception of the condition of the healthcare sector and its concepts on care, and also assistance in decision-making via the design of the common condition into action are some of the purposes of creating dashboard visualizations in healthcare [38].

Khan and Khan [42] tipped to use of visual techniques of data including tables, pie chart, bar graph, histogram, line graph, area charts, scatter charts, bubble charts, and multiple data series. The use of visualization techniques include parallel coordinates, map tree, entity-relationship diagram, coniferous trees, timeline, flow charts, data flow diagrams, Venn diagrams, and semantic network and also using the mechanism of interaction, including zooming in and out, outline, and detail are important aspects. Helping people to understand the data and focusing on evaluation or analysis, providing visual data to understand the most effective information, are the functions of dashboards.

Information visualization can be used as a useful tool to transmit insights into data and also as a tool for relationship and cooperation [43]. Yigitbasioglu and Velcu [44] consider principles like the possibility of changing the formats of displaying information, the possibility of pop-up and automated alerts, the ability to drill down and drill up, the possibility of integration to online analytical processing system or data warehouse, single page display and using color and guidelines to design in two-dimensional and three-dimensional diagrams, and zoom in and zoom out. These principles make flexibility of the dashboards to leverage the strategy and corporate values.

Gröger et al. [45] point to the three-tier architecture including data security, data analysis, and announcement of results and presentation layer and know their results comprehensive data warehouse with processing and operational data and providing data near real time, calculation criteria, storage of pattern recognition based on data mining and open sharing of knowledge in audio and video communications, and intuitive and easy user interface, combined with customized content mobile and flexible access.

Because the physical and conceptual characteristics of system components are primarily considered by traditional human factors design procedures and principles, rather than the manner that the integrated system requires to function from a cognitive point of view, they are not adequate for accessing the situation consciousness required in complicated systems [39]. References [46, 47] stated that we require cognitive the science of processing data for storage and retrieval, with its insights consideration the complicated the department of healthcare work, which is concreted with the principles of human-centered design for dashboard systems that support human understanding of the apply and use of information via health information technology [38]. Similarly, the healthcare activities and processes must be understood and recognized in order to understand the dangers and also the necessary supports for the consciousness of the situation [38].

Karami [48] mentions principles such as determining the purpose of dashboard design and coordination with organizational goals, determining the key performance indicators, set a time frame, extracting detailed data, flexibility, drilling down and analysis capabilities, security, how to display, displaying a warning, and knowing their results. Also the author defined goals and how they meet, design appropriate to the objectives and vision of the organization, specific measures to improve the quality of performance, updated information according to user view, type of use and the importance of the task, relevant and accurate data to standard definitions and acceptable to calculate, optimal functionality and personalization based on user requirements are the other principle. He points to the ability for users to perform deep analysis by clicking on operational indicators, protect data security according to the visual design components, and presentation, highlighting important information as critical values.

Cahyadi and Prananto [49] point to principles such as possibility of drilling down, selecting the main criteria, access to clear and reliable data, database technology, adequate infrastructure and data warehouse for the organization, and ability to analyze and predict. They consider the benefits of these principles as follows: users are encouraged and become consulting and propagated the use of different types of reports and forecasting models and also dashboards, and see the information in a wider perspective. According to the specific needs of user's level, elaborated information which is presented to different levels is customized. Based on criteria like interaction with the dashboard, amount of data displayed to users at different levels and ensuring the process of merge, integration, and standardization of data, dashboards can be considered successful and effective.

Mattingly et al. [50] point to the flexibility design to support changing project requirements, real-time capability, easy development, and maintenance and consider them useful for improving organizational behavior.

Rouhani et al. [10] designed a hospital dashboards based architectural framework and surveyed the satisfaction of those dashboards through end-user computing satisfaction (EUCS) model and concluded in the middle of the variables that the highest satisfaction was related to the format and the least satisfaction among the users transmitted the accuracy aspect.

## 3. Methodology

In this study, first, the metasynthesis qualitative research method was utilized to extract guiding principles of dashboard architecture through the review of credible corporate dashboards and studies of different data sources in the dashboard scope. The resulting principles and framework are needed to design and architect the dashboard; then by the comparative approach, the current research results are matched by studying related works.

The metasynthesis is a qualitative study that reviews extracted information and findings from other qualitative studies with the related issue. As a result, the sample for metasynthesis will be from selected qualitative studies and based on their relevance to the research question [51].

According to [52], metasynthesis involves seven steps, including setting the research questions, conducting systematic literature, search and selection of suitable articles, extracting information of articles, analysis and composition of the qualitative findings, quality control, and presentation of results. In the third step of the metasynthesis method including search and selection of suitable articles, qualified remaining articles will be evaluated through the critical evaluation method and articles are ranked in terms of quality. Finally, the remaining articles for extracting the required data will be the fourth step of the metasynthesis method. Critically evaluating is a systematic method for checking the searched articles, where the basic characteristics of each research article as fair and objective are examined. In the meantime, what will be assessed is the validity and relevance of the article.

The statistical population is resources available in the dashboard. The statistical sample was chosen with the purposive sampling method from the statistical population.

In the present study for analyzing the quality findings used of the encryption method, encryption refers to the process of analysis which diagnosed the concepts and discovered their dimensions and characteristics in the data. In this way of encryption, the code is extracted from the text and then this extracted code is encrypted again that this forms concepts and finally does other types of encryption on the implications that result in categories. In the analysis, there is open, axial, and choice encryption. After the open encryption process, the data are divided into concepts and classifications; axial encryption linked them together to show their relationship and categories and subcategories in the new form. It is the time that classification had to be only a general theoretical scheme. So after axial encryption, selective encryption is done. Selective encryption is integration and correction theory.

In the metasynthesis method, saturation and refining will be used. Unlike random sampling, in which the goal is to generalize the results of a representative sample of the population studied, this goal is not considered in qualitative methods and criteria are to describe or explain phenomena in detail as possible. Therefore, the introduced criteria to maximize the information about the events are considered as the endpoint. The benchmark in the field of qualitative research is called saturation. This occurs when no more data to develop, modify, enlarge, or add to the the existing theory are found [53]. In this situation, the new data to be classified into the existing research does not change or does not propose to create a new category [54].

One of the most important steps in conducting a systematic review of metasynthesis is the formulation of standards for the reception of articles for use in the next steps of metasynthesis and also defining the criteria for rejection of articles of this process, in order to refine them.

## 4. Results

In this study, a metasynthesis as a method is utilized to achieve a comprehensive mix of design principles, based on a translation of limited qualitative studies.

In the first step of this procedure, the most creative questions with interrogative words that are common in scientific research are created as follows:

- What: principles and guidelines for designing enterprise dashboards.
- What: principles and guidelines for the technical architecture enterprise dashboards.
- Who: the study population included international resources available in the dashboard.
- When: the time frame investigated in this study is from 2010 to 2016.
- How: in the method used to collect data in this study, secondary data have been used to name past documents. These documents include all of the researches (including research and review) in the field of principles of design and technical architecture for organizational dashboards. This data collection is famous for the documentary analysis. In metasynthesis addition to the findings, past research text (including review and research) is as data.

In the second step, with a systematic search in the repository of published articles, the right keywords related to the topic were selected and quested. Downloading the full text is completely based on keywords and study of each article adds to keywords. After adding new keywords, research is necessary in order to complete the investigation. Some of the keywords used are Dashboard, Enterprise, Guideline, Framework, Decision support, KPI, and so on. 2010 to 2016 timeframe will be evaluated throughout the study. Also, browsing and resources of each of the articles must be checked (check backward documentation) and some articles on topics related to the research questions are extracted from scientific databases. Some of the databases used are Springer, ScienceDirect, IEEE, Wiley, Emerald, and so on. After the investigation of databases using keywords and reviewing the title of articles and also checking the reference lists of downloaded articles and attain a state of saturation, the number of 78 articles and 24 books was finalized.

In the third step, the found resources in the previous step for step by step in stages are evaluated and refined. In metasynthesis, acceptance criteria and rejection criteria are used for the selection of suitable articles and deleting unsuitable articles.

Acceptance and rejection criteria used in this study are shown in Table 1.

In the review, the process researcher determines which of the articles are according to the research question and which should be discarded. In order to achieve this goal, articles have been revised several times and during the review, some of them are excluded. Therefore, during this process, articles have been refined and their number reduced gradually. Finally, the remaining number of resources for use in the next step of the metasynthesis method is the sample size of 12 articles out of 102 articles.

Selected articles using the acceptance and rejection criteria are shown in Table 2.

In this study, after reviewing the literature and their ratings according to criteria of the critical evaluation method, one article in terms of quality was evaluated very good, 10 papers were evaluated good, and a paper was evaluated medium; they are shown in Table 3.

In the fourth step, selected and final resources have been fully studied again. Through examining them, the dimensions of principles and guidelines for design and architect of enterprise dashboards are extracted from findings of the scientific resources.

In the fifth step, with the name of analyzing, the open, axial, and choice coding have been applied. In the initial phase, open coding, dimensions, indexes, and subindexes of principles and guidelines for design and architect of enterprise dashboards, extracted and classified from findings of articles and to each of the indicators and subindicators, were assigned the code.

In the second phase with the name of axial coding: codes that had overlapped were identified, overlaps were eliminated, and codes that had common contents were detected. Defined common codes which are the outputs of this stage are 15 main indicators and 66 secondary indicators. Identification codes are examined, and the codes associated with each of the subindices were in a group.

In this study, 66 subindexes in the 15 groups and in five main dimensions, entitled “Principles and guidelines for design and technical architecture of enterprise dashboards” were categorized: objectives and rules, user interface, data processing and analysis, data architecture and technical requirements, and functions.

In the third phase with name of selective coding: identified principles and guidelines were classified in the framework of “Multilayer System Architecture.” These layers include the presentation layer, application layer, data layer, technical infrastructure layer.

Maintaining the quality of the projects is essential in the sixth step; therefore every step of the metasynthesis method should have a strong argument. Acceptable techniques, techniques accepted in the scientific community, manual and electronic search methods, and extraction articles and results should be observed in this stage.

In the final step, principles and guidelines for the design and technical architecture of enterprise dashboards obtained with the metasynthesis method were in the form of layers of system architecture as shown in Table 4.

## 5. Conclusion

Subsequently studying the dimensions and indicators of principles or guidelines for design and architect of enterprise dashboards extract from findings of articles, they are transparent through comparing with related works. For example, [55] determines the best approach for designing general health dashboards and suggests an optimized user interface for emergency response system for government public health laboratories. Therefore according to the desired scope, factors such as display all indicators in one screen without the need to move the other pages, using charts and graphs in the right place for visualization and interpretation to minimize the decision-making time and also deploying analytics methods are organizational benefits of dashboards. Therefore, in accordance with the principles obtained in this study, they pointed out the principles and guidelines of interaction and how to view the presentation layer, analysis and forecasting of the application layer, and maintenance of the technical infrastructure layer.

Table 5 illustrates previous studies which are compared by current research in extracted indicators. As can be concluded in, [45, 48] , most of extracted indicators in this study are analogous with related works, although the contribution of this research is categorizing principles and indicators in healthcare industry and mapping them in the form of multilayer architecture.

The contribution of the current work is contrary to other works, which is listing and classifying aspects of the architectural principle. The following is done in order to answer the research question, “The principles and guidelines for design and technical architecture a convenient dashboard means?” A review of the literature and studies from different data sources in the dashboard era was done and also by utilizing the steps of the metasynthesis, principles, and guidelines for the design and architecture of enterprise, dashboards were classified as “Multilayer System Architecture”. In this study, offering an elaborated and comprehensive framework for dashboards design has been done which distinguishes it from other studies in the area of dashboards.

According to the prescribed timeframe 2010 to 2016 and also the Persian and English language of articles in the acceptance criteria of the research method, the omitted sources were a limitation of this study.

It is recommended for future research that the category of principles and guidelines for design and architect of enterprise dashboards should be investigated in the form of layers except multilayer architecture and this study is to be done in an expanded time period and in different languages.

## Figures and Tables

**Table 1:** Acceptance and rejection criteria.

	Rejection criteria	Acceptance criteria
Language of research	Except for Persian and English	Persian and English
Time of studies	Before 2010	From 2010 to 2018
Methods of study	Nonqualitative methods	Qualitative methods to collect and analyze data
The population of study	Except for enterprise dashboards	Enterprise dashboards
The conditions of study	Except for principles and guidelines for design and technical architecture of enterprise dashboards	Principles and guidelines for design and technical architecture of enterprise dashboards
Type of study	Personal views and articles invalid	Articles published in journals and conferences

**Table 2:** Selected articles.

Author	Title	Journal	Year
Hansoti	Business Intelligence Dashboard in Decision Making	Technology	2010
Mohd, Embong, and Zain	A Framework of Dashboard System for Higher Education Using Graph-Based Visualization Technique	Communications in Computer and Information Science	2010
Kuo, Tsai, and Kang	A framework of information visualization for multi-system construction	Automation in Construction	2011
Pappas and Whitman	Riding the technology wave: effective dashboard data visualization	Lecture Notes in Computer Science (including subseries Lecture Notes in Artificial Intelligence and Lecture Notes in Bioinformatics)	2011
Elias and Bezerianos	Exploration views: understanding dashboard creation and customization for visualization novices	Lecture Notes in Computer Science (including subseries Lecture Notes in Artificial Intelligence and Lecture Notes in Bioinformatics)	2011
Khan and Khan	Data and information visualization methods, and interactive mechanisms: A survey	International Journal of Computer Applications	2011
Yigitbasioglu and Velcu	A review of dashboards in performance management: Implications for design and research	International Journal of Accounting Information Systems	2012
Kintz	A semantic dashboard description language for a process-oriented dashboard design methodology	CEUR Workshop Proceedings	2012
Gröger et al.	The Operational Process Dashboard for Manufacturing	Procedia CIRP	2013
Lechner and Fruhling	Towards Public Health Dashboard Design Guidelines	International Conference on HCI in Business	2014
Karami	A Design Protocol to Develop Radiology Dashboards	Acta Informatica Medica	2014
Cahyadi and Prananto	Reflecting design thinking: A case study of the process of designing dashboards	Journal of Systems and Information Technology	2015
Auliya, Aknuranda, and Tolle	A Systematic Literature Review on Healthcare Dashboards Development: Trends, Issues, Methods, and Frameworks	Advanced Science Letters	2018

**Table 3:** Selected articles rating based on critical evaluation method.

	Hansoti	Mohd, Embong, and Zain	Kuo, Tsai, and Kang	Pappas and Whitman	Elias and Bezerianos	Khan and Khan	Yigitbasioglu and Velcu	Kintz	Gröger et al.	Lechner and Fruhling	Karami	Cahyadi and Prananto	Auliya, Aknuranda, and Tolle
Research purposes	3	4	4	3	3	4	4	3	4	4	4	4	4
Logic method	3	4	4	3	4	4	4	3	4	3	4	4	4
Research plan	4	4	4	3	4	3	3	3	4	3	4	4	5
Sampling	3	4	2	3	4	4	4	2	4	4	4	4	4
Data collection	3	4	3	3	4	4	4	2	4	4	4	4	3
Reflectivity, including the relationship between the researcher and the participants are	4	4	4	4	4	4	4	4	4	4	4	4	4
Ethical considerations	4	4	4	4	4	4	4	4	4	4	4	4	4
Carefully analyze the data	4	4	4	3	4	4	4	4	4	3	4	4	3
Articulate findings	3	4	4	3	3	4	4	3	3	3	4	4	4
The value of research	3	4	4	3	3	3	4	2	3	3	4	5	5
Total points	34	40	37	32	37	38	39	30	38	35	40	41	40
	Good	Good	Good	Good	Good	Good	Good	Medium	Good	Good	Good	Very good	Good

**Table 4:** Principles and guidelines for design and technical architecture of enterprise dashboards obtained with metasynthesis method.

Layers of system architecture	The main principles	Subsidiary principles and guidelines for design and technical architecture of enterprise dashboards
Presentation layer	Q1: target	SQ1goal setting dashboard, SQ2 according to the type of dashboard (strategic, analytical, and operational), SQ3 match data types with the goals of dashboard, SQ4 harmony with the goals and vision of the organization, and SQ5 monitoring process
	Q2: organizational culture	SQ5 attention to corporate culture to technology adoption
	Q3: type and user personality	SQ6 depend on the effectiveness of each of the principles to the needs of different parts of the organization, SQ7 regarding the objectives, terms and requirements of users, personality analysis users interacting layers of dashboard, SQ8 support from the local language, provide detailed explanations about the functioning of dashboard, and SQ9 view detailed information to users according to the profile, background, experience, efficiency, skills, and particular needs of any user at any level of executive, management, and operational
	Q4: interaction	SQ9 interactive functions discovery information, highlighting important information such exceptions, controllers time and data extraction, SQ10 zoom in and zoom out, Outline and detail and fisheye technique, SQ11 change the display size and location information according to the importance, SQ12 move the items and rotate it, SQ13 possible to drill down and drill up, SQ14 slices Dice, SQ15 filtering capabilities partial and total data, SQ16 possibility of changing the formats of display information, such as graphs and tables, SQ17 possibility of pop-up and control commands and warning, SQ18 links to related information, SQ19 possible clipboard and labeling and note documentation (metadata) for charts, SQ20 ability to group data and selection criteria, SQ21 open sharing of knowledge for audio and video communications and sending messages, SQ22 use the map to locate, and SQ23 reports in Word and PDF
	Q5: how to view	SQ24 four types of display time information, hierarchical, relational and multidimensional, SQ25 possibility selecting shared information in a variety of other displays, SQ26 opportunity to display different colors in the different time and show important information, SQ27 use the guidelines in the design charts of two-dimensional and three-dimensional, SQ28 possible to compare the data with line charts, bar, spot, scatter, bubble, SQ29 display information in a page without having to scroll page, SQ30 visual distinction clear between data that were selected and those that filter were, SQ31 techniques of visualization of data tables, pie charts, bar, histogram, line, area, scatter, bubble and a series of multiple data, SQ32 methods of visualization data coordinates: parallel, tree map, entity-relationship diagram, coniferous tree, timeline, flow diagrams, data flow, van and semantic network, and SQ33 displayed based on time priority, urgency, and effectiveness
Application layer	Q6: determine indicators	SQ34 determine the appropriate Key Performance Indicators and SQ35 index changes due to user interaction
	Q7: analysis and forecasting	SQ36 data mining, clustering and analyzing the results, SQ37 calculation criteria, SQ38 storage pattern recognition based on data mining, scenario analysis, SQ39 full access of users to data components for dimensional analysis and OLAP, SQ40 techniques to analyze time trends and Viewing past data, SQ41 aggregated data to analyze and interpret data correctly, SQ42 appropriate structure of the data warehouse for data mining, online analytical processing and knowledge extraction, and SQ43 ability to analyze and predict the effects of decisions
	Q12: accessibility	SQ58 web access; SQ59 mobile access
	Q13: privatization	SQ60 flexibility and optimal functionality and personalization based on user requirements, organization, and changed terms
Data layer	Q11: database	SQ50 data processing layer is responsible for extracting the data from data warehouse to update the necessary information, SQ51 supplies data regarding the type of dashboard (strategic, analytical, and operational), SQ52 methodology for process monitoring and data warehouse engine, SQ53 data providing system ERP, SQ54 data warehouse integrated with process data and operational security and data close to real-time SQ55 ETL process for the extraction of data warehousing, data mining of relevant and accurate standard definitions and acceptable to calculate, SQ56 data sources standard for sharing, date Science and better queries from them, and SQ57 access to clear and reliable data from enterprise multiple sources
Technical infrastructure layer	Q8: system architecture	SQ44 according to the architect defined for the system
	Q9: infrastructure	SQ45 proper design of data warehouse and data collection of systems, SQ46 according to build reports algorithms, network, relational database, relationships between systems, and SQ47 database technology and adequate infrastructure and data warehouse for the organization
	Q10: integration	SQ48 enable integration with online analytical processing system and data warehouse or other systems and SQ49 different sources of data, merger, consolidation, standardization, and be related dashboard
	Q14: maintenance	SQ61 ability to change and update indicators, SQ62 possibility of debugging and correction and updating easy and flexible algorithms, SQ63 training and guidance in real time, and SQ64 set a time frame for updating information according to user, type of use, and the importance of duty
	Q15: security	SQ65 methods, techniques, and technologies used to protect data security and SQ66 attention to system security

**Table 5:** Extracted indicators with research that pointed to these indicators, in comparison with this study.

Extracted indicators	Hansoti	Mohd, Embong, and Zain	Kuo, Tsai, and Kang	Pappas and Whitman	Elias and Bezerianos	Khan and Khan	Yigitbasioglu and Velcu	Kintz	Gröger et al.	Lechner and Fruhling	Karami	Cahyadi and Prananto	Auliya, Aknuranda, and Tolle	This study
	2010	2010	2011	2011	2011	2011	2012	2012	2013	2014	2014	2015	2018	
Target				**✓**			**✓**	**✓**			**✓**	**✓**	**✓**	**✓**
Organizational culture											**✓**	**✓**		**✓**
Type and user personality	**✓**	**✓**		**✓**	**✓**		**✓**		**✓**		**✓**	**✓**	**✓**	**✓**
Interaction	**✓**	**✓**	**✓**	**✓**	**✓**	**✓**	**✓**	**✓**	**✓**	**✓**	**✓**	**✓**	**✓**	**✓**
How to view	**✓**	**✓**	**✓**	**✓**	**✓**	**✓**	**✓**	**✓**	**✓**	**✓**	**✓**		**✓**	**✓**
Determine indicators		**✓**		**✓**			**✓**	**✓**	**✓**		**✓**	**✓**		**✓**
Analysis and forecasting		**✓**			**✓**	**✓**	**✓**		**✓**	**✓**	**✓**	**✓**	**✓**	**✓**
Accessibility	**✓**								**✓**		**✓**		**✓**	**✓**
Privatization	**✓**								**✓**		**✓**			**✓**
Database		**✓**	**✓**	**✓**				**✓**	**✓**		**✓**	**✓**	**✓**	**✓**
System architecture		**✓**	**✓**					**✓**	**✓**					**✓**
Infrastructure			**✓**								**✓**	**✓**		**✓**
Integration	**✓**						**✓**				**✓**	**✓**		**✓**
Maintenance		**✓**	**✓**					**✓**	**✓**	**✓**	**✓**			**✓**
Security	**✓**										**✓**			**✓**
